This article has been retracted.

# Human Umbilical Cord Mesenchymal Stem Cell-Derived Exosome Repairs Endometrial Epithelial Cells Injury Induced by Hypoxia via Regulating miR-663a/CDKN2A Axis

**DOI:** 10.1155/2022/3082969

**Published:** 2022-10-12

**Authors:** Hanbi Wang, Simiao Liu, Wanyu Zhang, Meizhi Liu, Chengyan Deng

**Affiliations:** Department of Obstetrics and Gynecology, National Clinical Research Center for Obstetric & Gynecologic Diseases, State Key Laboratory of Complex Severe and Rare Diseases, Peking Union Medical College Hospital, Chinese Academy of Medical Science and Peking Union Medical College, Shuai fu yuan, Dongcheng District, Beijing 100730, China

## Abstract

**Aim:**

Thin endometrium remains a severe clinical challenge with no effective therapy to date. We aimed at exploring the role and molecular mechanism of human umbilical cord mesenchymal stem cell- (hucMSC-) derived exosomes (hucMSC-Ex) in repairing hypoxic injury of endometrial epithelial cells (EECs).

**Methods:**

Exosomes were harvested from the conditioned medium of hucMSC and characterized using western blot, transmission electron microscopy (TEM), flow cytometry, and nanoparticle tracking analysis (NTA). EECs were subjected to hypoxic conditions before cocultured with hucMSC-Ex. Cell viability, apoptosis, and migration were determined with CCK-8, flow cytometry, and wound healing assay, respectively. Apoptosis/EMT-related proteins were detected by western blot. The miRNA profiling was determined by RNA sequencing. The expression of miR-663a and CDKN2A was measured by qRT-PCR. MiR-663a in EECs was overexpressed by transfecting with miR-663a mimics.

**Results:**

Mesenchymal stem cells (MSCs) markers CD73, CD90, and CD106 were positively expressed in hucMSCs. Exosome isolated from hucMSC expressed CD63 and TSG101, and were 100–150 nm in diameter. HucMSC-Ex promoted cell proliferation inhibited by hypoxia. And hucMSC-Ex also inhibited hypoxia-induced apoptosis, migration, and EMT of EECs by upregulating the expression of Bcl-2 and E-cadherin and downregulating Bax and N-cadherin levels. Further, bioinformatics research found that hucMSC-Ex coculture can significantly upregulate the expression of miR-663a and decrease the expression of CDKN2A in hypoxia-induced EECs. Furthermore, miR-663a overexpression inhibited CDKN2A expression and increased the expression of Bcl-2 and E-cadherin in hypoxia-induced EECs.

**Conclusions:**

HucMSC-Ex promoted cell proliferation, inhibited cell apoptosis, migration, and EMT in hypoxia-induced EECs, thereby alleviating hypoxia-induced EECs injury, which may be related to its regulation of miR-663a/CDKN2A expression. Our study indicated that hucMSC-Ex might benefit for repairing thin endometrium.

## 1. Introduction

Human endometrium is a highly dynamic renewable tissue which receives embryos by implantation during a woman's reproductive period [1]. Endometrial impairments initiated by infection, caesarean section, recurrent curettage, or myomectomy can result in thin endometrium [2]. It is reported that a thin endometrial lining is related to declined rates of implantation and pregnancy [3]. Hormone-therapy, vasoactive measures, intrauterine infusion of growth factor, and regenerative medicine are modalities offered for the treatment of thin endometrium [4], whereas clinical efficacy of these means is negligible. Hence, innovative strategies to rebuild the endometrium to its normal morphology and function are essential for treatment.

Mesenchymal stem cells (MSCs) are a particular stromal cell type which presents structural and functional benefits in diseases, such as thin endometrium [5]. The transplantation of MSCs has been studied as a scheme to regenerate the endometrium because of their capability to differentiate into endometrial stromal cells (ESCs) and endometrial epithelial cells (EECs) [6]. Accumulating evidence has demonstrated the therapeutic impacts of MSCs on endometrium, such as the increased endometrium thickness, better formed tissue construction, protected implantation, and ameliorated pregnancy [7]. Exosomes are potent secretory products of MSCs that play a crucial role in biological effects mediated by MSCs [8]. MSCs-derived exosomes reverse epithelial-mesenchymal transition (EMT) and facilitate repair of damaged endometrium [9]. Moreover, the local transplantation of umbilical cord mesenchymal stem cells- (UCMSCs-) derived exosomes (hucMSCs-Ex) loaded in collagen scaffold facilitates endometrium regeneration and promotes fertility restoration [10]. Exosome-shuttled miR-7162-3p from hucMSCs repairs ESCs injury [11]. In comparison with their source cells, exosomes display the advantages of easier storage, easier perfusion into tissues, immune-privileged status, and higher biological stability [12]. Therefore, exosome-based therapeutic strategies hold promise as a prospective approach to promoting endometrial regeneration.

MicroRNAs (miRNAs), posttranscriptionally controlling the translation and stability of mRNAs, are a crucial component of the exosomal cargo [13]. It has been proved that exosome-encapsulated miRNA can be stored stably to avoid nuclease degradation [14]. miR-663a is reported to be able to suppress early apoptosis and stimulate proliferation of human spermatogonial stem cells [15]. MiR-663a is found to be associated with the development of renal cell carcinoma, which promotes cellular proliferation and migration while inhibiting apoptosis [16]. Cyclin-dependent kinase inhibitor 2A (CDKN2A, also known as p16 gene, which is located on chromosome 9P21) is the first antioncogene directly involved in cell cycle regulation [17]. CDKN2A protein competes with cyclin-dependent kinases 4/6 (CDK4/6) to inhibit its activity, inducing cells to stop in G1 phase, thereby inhibiting cell proliferation [18]. CDKN2A is reported to mediate the development of the disease by regulating apoptosis [19, 20]. Online software predicts the binding relationship between miR-663a and CDKN2A. However, a relationship between the anti-injury effect of MSCs-derived exosomes on EECs in hypoxic conditions and miR-663a regulation of CDKN2A has not been established.

Therefore, we hypothesized that MSCs-derived exosome are involved in regulating apoptosis and migration in EECs under hypoxic injury environment through miR-663a. We further investigated the potential target of exosomal derived from hucMSCs in attenuating EECs apoptosis and migration.

## 2. Materials and Methods

### 2.1. EECs and hucMSCs Cell Culture

Primary human EECs were bought from iCell Bioscience Inc. (HUM-iCELL-f004, China) and cultured in Dulbecco's modified Eagle's medium (Gibco, 11965092, America) with 10% fetal bovine serum (Gibco, 10100147, America). hucMSCs at passage 3 were obtained from iCell Bioscience Inc. (HUM-iCell-e011, China), and they were maintained in DMEM/F12 (Gibco, A4192001, America) containing 10% exosome-depleted FBS (Gibco, A2720801, America). As previously described, hucMSCs at passage 4–6 were applied for the subsequent experiments. 100 ng/ml penicillin and 100 U/ml streptomycin were added in the culture medium, and cells were then maintained in normoxic (21% O_2_, 75% N_2_, and 5% CO_2_) condition at 37°C. Cells were stained by immunofluorescence to determine their purity after 24 h of culture.

### 2.2. Identification of hucMSCs

The phenotype profile of hucMSCs was evaluated through flow cytometry analysis by using antibodies against positive markers (CD73, CD90, and CD105) and negative markers (CD14, CD34, and CD45). All details of antibodies are shown as follow: fluorescein isothiocyanate- (FITC-) conjugated antibodies against CD73 (BioLegend, 344016, America), CD105 (BD, 562351, America), CD90 (BioLegend, 328108, America), phycoerythrin- (PE-) conjugated antibodies against CD34 (BD, 348057, America), CD45 (BD, 560975, America), and CD14 (BD, 567731, America).

### 2.3. Harvest and Characterization of HucMSC-Ex

Exosomes were separated from hucMSCs as previously described [21]. The separation procedure included an additional centrifugation step to remove small cell debris prior to ultracentrifugation for 1 h at 100,000 g to generate an exosome pellet. Next, PBS was used to resuspend the pelleted exosomes. Exosomal markers including TSG101 (Abcam, ab125011, UK) and CD63 (Abcam, ab134045, UK) were used for western blot. The morphology of exosomes was observed under transmission electron microscopy (TEM). The size distribution of exosomes was examined by nanoparticle tracking analysis (NTA) [10]. The concentration of exosomes was determined using bicinchoninic acid (BCA) protein kit (Thermo, 23227, USA).

### 2.4. EECs Hypoxia Injury Model and Grouping Treatment

EECs were cultured in normoxic condition and grown to approximately 60–70% confluence. EECs incubated in normoxic condition were used as control, named as the normal group. For hypoxia treatment, cells were cultured under humidified hypoxic air (1% O_2_, 94% N_2_, and 5% CO_2_) in a modular incubator chamber (Thermo, America) at 37°C for indicated periods (1 h, 4 h, 8 h, 16 h, and 24 h), named as the hypoxia group. Hypoxia injury of EECs was evaluated by western blot. Hypoxia-induced EECs (1 × 10^5^/per well) was cocultured with 2 *μ*g of hucMSC-Ex on the basis of protein measurement, named as the hypoxia+hucMSC-Ex group.

### 2.5. PKH67 Labeling

Exosomes from hucMSCs were labeled with PKH67 (Sigma-Aldrich, MINI67-1KT, Germany) in accordance with the protocol. After incubation with PKH67-labeled exosomes for 24 h, EECs were fixed with paraformaldehyde (4%), permeabilized with Triton X-100 (0.5%), and stained with DAPI. Afterwards, a laser scanning confocal microscope (Olympus FLUOVIEW FV3000) was used to detect the uptake of labeled exosomes by EECs.

### 2.6. CCK-8 Assay

The cell counting kit 8 (Beyotime Biotechnology, C0038, China) was used to measure cell viability. EECs were seeded in 96-well plate and cocultured with or without hucMSC-Ex for 24 h. Next, cells in each well were added with CCK-8 reagent (Solarbio, China) and incubated for 2 h at 37°C. OD value was measured with a microplate reader (molecular devices-spetramax paradigm) at 450 nm.

### 2.7. Cell Apoptosis

EECs were planted in 6-well plate (5 × 10^5^ cells/well) and cocultured with or without hucMSC-Ex for 24 h. The annexin V-fluorescein isothiocyanate (FITC)/propidium iodide (PI) apoptosis detection kit (Beyotime Biotechnology, C1062, China) was used to determine apoptosis according to the manufacturer's guidelines. Cells were sorted within 1 h by a FACScan flow cytometer (BD FACS Calibur).

### 2.8. Wound Healing Assay

EECs were planted in 6-well plate in culture medium and grown to confluence. A sterile 200 *μ*l pipette tip was utilized to scratch the monolayer of exposed EECs. Cells were rinsed by PBS prior to incubating in fresh medium. At 0 h and 24 h, wounds were imaged under phase-contrast microscopy. Subsequently, wound closure was evaluated and showed as the percentage of closure regarding initial wound width.

### 2.9. qRT-PCR

Total RNA was extracted from EECs using RNAzol® RT kit (Sigma-Aldrich, R4533, Germany), cDNA of mRNAs was synthesized by Prime Script™ RT reagent (TIANGEN BIOTECH, KR118, China), and cDNA of miRNA was synthesized by TransScript® miRNA First-Strand cDNA Synthesis SuperMix (TransGen Biotech, AT351, China). SYBR® Premix Ex Taq™ (Tli RNaseH Plus, FP205, China) were applied to determine the relative levels of target genes. StepOnePlus Real-Time PCR System (ABI 7500 Fast) was used to perform real-time PCR procedure. U6 and GAPDH were used as the internal reference. The RNA expressions were quantified and calculated with the 2^−ΔΔCt^ method. Primers are shown in Table 1.

### 2.10. Western Blot

Total proteins of cells were extracted with RIPA lysis buffer (25 mM Tris-HCl (PH7.4), 150 mM NaCl, 1% NP40, and 0.25% sodium deoxycholate) and separated with 10% SDS-polyacrylamide gel electrophoresis (SDS-PAGE), followed by transferred onto polyvinylidene fluoride (PVDF) membranes (Sigma-Aldrich, IPFL00010, Germany). Membranes were incubated in primary antibodies at 4°C overnight including CD63 antibody (Abcam, ab134045, UK), TSG101 antibody (Abcam ab125011, UK), VEGF antibody (Abcam, ab214424, UK), av*β*3 antibody (Abcam, ab179473, UK), CDKN2A/p16INK4a antibody (Abcam, ab108349, UK), Bax antibody (Abcam, ab182734, UK), cleaved-caspase3 antibody (Abcam, ab32042, UK), P53 antibody (Abcam, ab26, UK), Bcl-2 antibody (Abcam, ab182858, UK), E-cadherin antibody (Abcam, ab40772, UK), N-cadherin antibody (Abcam, ab76011, UK), *β*-actin antibody (Cwbio, CW0096, China), and *β*-tubulin antibody (Cwbio, CW0098, China). After incubation with secondary antibodies (ZSGB-BIO, China), protein signals were measured and visualized with an ECL chemiluminescence kit (Cytiva, RPN2232, China) under a luminescent imaging system (CIiNX ChemiScoe 6100).

### 2.11. miRNA Sequencing

After being extracted from cells, the quality of the total RNA was examined with an Agilent Technologies 2100 Bioanalyzer. TruSeq small RNA library prep kit (RiboBio, China) was applied to prepare the small RNA library. After multiplexed in equimolar amounts, indexed small RNA libraries were denatured and loaded for cluster generation on GAIIx flow cell lanes with cBot station and Illumina cluster generation kits. Differentially expressed miRNAs presenting raw reads ≥5 in samples and *P* value <0.05 were selected. The target genes of identified miRNAs were predicted using miRNA target prediction algorithms TargetScan (https://www.targetscan.org/vert_80/) [22].

### 2.12. Cell Transfection

miR-663a mimics (miR-663a mimics) and mimics NC (NC) were synthesized by Sangon Biotech (Shanghai) Co., Ltd., before transfection, EECs (2 × 10^4^/well) were seeded in 6-well plates and grown to 80% confluence. miR-663a mimics and mimics NC (final concentration: 30 nM/well) were transfected into EECs using transfection jetPRIME® (Polyplus, 114-15, France). Cells were incubated in normoxic or hypoxic condition for 4 h prior to collected for the subsequent detections.

### 2.13. Statistical Analysis

Data were analyzed and visualized using GraphPad Prism 6.0 and presented as mean ± standard deviation (SD). Significant differences between the two groups were determined by student's *t*-test. While one-way ANOVA analysis followed by Tukey's post hoc was carried out to compare the differences among more than two groups. *P* < 0.05 was considered statistically significant.

## 3. Results

### 3.1. Characterization of hucMSCs and hucMSC-Ex

First, we identified the surface antigens of hucMSCs. The surface antigens of hucMSCs were detected by flow cytometry, which presented that the negative markers (CD14, CD45, and CD34) were almost no expressed, while the positive markers (CD73, CD90, and CD105) for MSCs were highly expressed (Figures 1(a)–1(f)).

Next, we extracted exosomes from hucMSCs culture medium. Western blot showed that typical positive markers (TSG101 and CD63) were expressed in the isolated exosomes (Figure 2(a)). TEM imaging exhibited that the vesicle-like exosomes were spherical (Figure 2(b)). Moreover, NTA results revealed a narrow size distribution of exosomes, and the main peak was at 100-150 nm (Figure 2(c)). These data indicated that the purified exosomes were successfully extracted from the culture medium of hucMSCs.

### 3.2. HucMSC-Ex Promoted EECs Survival under Hypoxic Condition

To investigate the potential of hucMSC-Ex on thin endometrium, EECs were exposed to a hypoxic environment to establish a cellular model. With increasing incubation time under hypoxia condition, the protein expression of hypoxia-related proteins VEGF and av*β*3 were increased in EECs, while the level of epithelial marker E-cadherin was decreased (Figures 3(a)–3(d)). To verify the uptake efficiency of hucMSC-Ex by EECs, we cocultured hypoxia-induced EECs with PKH67-labeled hucMSC-Ex for 24 h. Compared with the normal group, the uptake of hucMSC-Ex by EECs cells in the hypoxia group was significantly increased (Figure 3(e)).

To further explore the function of hucMSC-Ex in cell proliferation in hypoxic-induced EECs, hypoxia-induced EECs were cocultured with hucMSC-Ex. Cell proliferation of EECs was reduced in hypoxic-induced EECs, which can be elevated after coculture with hucMSC-Ex (Figure 3(f)). The findings suggested that hucMSC-Ex promoted the cell survival of hypoxic-induced EECs.

### 3.3. HucMSC-Ex Inhibited Hypoxia-Induced Apoptosis, Migration, and EMT of EECs

Then, we further explored the role of hucMSC-Ex in cell apoptosis, migration, and EMT of hypoxia-induced EECs. The results showed that cell apoptosis in EECs with hypoxia treatment for 4 h was significantly increased compared with that in normoxic condition-incubated EECs, while apoptosis in hypoxia-induced EECs was significantly inhibited after treatment with hucMSC-Ex (Figures 4(a) and 4(b)). Moreover, compared with the normal group, hypoxia treatment promoted EECs migration, while hucMSC-Ex treatment significantly inhibited cell migration in hypoxia-induced EECs (Figures 4(c) and 4(d)). The promoted apoptosis of EECs under hypoxic condition was also evidenced by the elevated proapoptotic proteins (Bax, cleaved-caspase3, and P53) and downregulated Bcl-2. Besides, the enhanced migration of EECs induced by hypoxia was supported by the elevated mesenchymal biomarker N-cadherin and decreased epithelial marker E-cadherin, suggesting that hypoxia promoted EMT of EECs. However, hucMSC-Ex treatment reversed the protein expressions in EECs induced by hypoxia (Figures 4(e)–4(j)). Collectively, the data revealed that hucMSC-Ex inhibited cell apoptosis, migration, and EMT in hypoxia-induced EECs.

### 3.4. HucMSC-Ex Increased miR-663a in Hypoxia-Treated EECs, and miR-663a Negatively Modulated CDKN2A Expression

To explore differential expression miRNAs (DEmiRNAs) in EECs after treatment with hypoxia or hucMSC-Ex, miRNA sequencing analysis was performed. The results showed that 45 (36 upregulated and 9 downregulated) DEmiRNAs were identified in hypoxia, normal, and hypoxia+hucMSC-Ex groups (Figure 5(a)). Among that, miR-663a was significantly downregulated in hypoxia treated EECs, while its expression recovered after coculturing with hucMSC-Ex (Figure 5(b)). The mRNA expression of miR-663a was also validated with qRT-PCR (Figure 5(c)). We speculated that miR-663a in hucMSC-Ex exerted a protective effect on hypoxia-induced EECs. The online website TargetScan predicted that miR-663a could bind to CDKN2A 3′-UTR, and the targeting sequence was shown in Figure 5(d). We found that the expression of CDKN2A was upregulated in hypoxia-induced EECs, which was decreased after hucMSC-Ex coculture (Figure 5(e)). Then, we upregulated the miR-663a expression in hypoxia-induced EECs by transfecting with miR-663 mimics (Figure 5(f)). After transfection with miR-663a mimics, CDKN2A, N-cadherin, and Bax were downregulated, while antiapoptosis protein Bcl-2 and epithelial marker E-cadherin were both upregulated in hypoxia-induced EECs (Figures 5(g)–5(l)). The data indicated that CDKN2A could be negatively modulated by miR-663a. In addition, the effects of miR-663a overexpression was consistent with that of hucMSC-Ex coculture.

## 4. Discussion

MSCs have acquired much interest in the therapy of many disorders, which also displayed better protection in the treatment of thin endometrium [23]. Currently, MSCs-derived exosomes have been noticed to contain many kinds of mediators including proteins and miRNAs, mediating the function of MSCs [9, 24]. Moreover, the altered levels of miRNAs reported in thin endometrium indicate that miRNAs may be involved in the pathogenesis of this disorder [25]. Therefore, we investigated the function of hucMSC-Ex in EECs within hypoxic conditions. Collectively, this study demonstrated that hucMSC-Ex could indeed suppress EECs apoptosis and migration through regulating the miR-663a/CDKN2A axis.

MSCs are widely applied in the repair of damaged tissues [26]. MSCs can play its biological roles in repairing damaged tissues through secreting exosomes [27]. For instance, exosomes derived from bone marrow mesenchymal stem cells (BMSCs) can reverse EMT in EECs and are implicated in repairing the induced endometrium [9]. Exosomal transfer of BMSCs-derived miR-340 attenuates endometrial fibrosis [28]. Exosomes derived from hucMSCs promote proliferation of allogeneic ESCs [29]. hucMSCs-derived exosomal miR-7162-3p reduces ESCs apoptosis induced by mifepristone [11]. Exosomes derived from hucMSCs can improve cell viability and exhibit anti-inflammatory properties in EECs induced by oxygen and glucose deprivation/reoxygenation (OGD/R) [30]. HucMSC-Ex enhances the migratory ability of endometrial glandular epithelial cells isolated from endometriosis patients via promotion of EMT [31]. Collagen scaffold/UCMSCs facilitates endometrial regeneration and fertility restoration, in addition, better collagen remodeling, obvious luminal structures, and thicker endometrium are noticed [10, 32]. Importantly, MSCs can play an antiapoptosis role in disorders including cerebrovascular disease [33], cardiovascular disease [34], and reproductive disorder [13]. Transplantation of MSCs-derived exosomes can inhibit apoptosis and promote proliferation and migration in endometrial cells, thus improving endometrial repair [11, 29, 35]. On the basis of these discoveries, we proposed that MSCs-derived exosomes could be employed in thin endometrium therapy. In our cellular model of thin endometrium, we found that the number of viable EECs in hypoxic condition decreased and apoptosis and migration increased, whereas apoptosis and migration inhibited by coculture with hucMSC-Ex. In EECs under hypoxic condition, the elevated proapoptotic proteins and downregulated antiapoptotic protein were observed. Besides, migration related proteins N-cadherin and E-cadherin were increased and decreased, respectively. After treatment with hucMSC-Ex, the number of viable EECs within hypoxia condition was increased, while apoptosis and migration were inhibited. Thus, hucMSC-Ex exerted a protective effect on hypoxia-induced EECs injury.

Further, we screened differentially expressed miRNAs in EECs following hypoxia or hucMSC-Ex treatment by RNA-seq. It was found that miR-663a was significantly downregulated in hypoxia-induced EECs, while its expression was restored after coculture with hucMSC-Ex. This result was also validated by qRT-PCR. A previous study shows altered expression of miR-663a associated with hypoxia in bronchoalveolar lavage fluid [36]. miR-663a can suppress early apoptosis and stimulate proliferation of human spermatogonial stem cells [15]. miR-663a stimulates cell proliferation and migration in osteosarcoma [37]. In addition, bioinformatics analysis predicted that miR-663a could target CDKN2A 3′-UTR. Studies showed that apoptosis and proliferation are intimately coupled. Many proteins and signal pathways have been proved to play key role in cell proliferation and apoptosis, such as c-Myc, p53, pRb, Ras, PKA, PKC, Bcl-2, NF-*κ*B, CDK, cyclins, CKI, and MAPK/ERK, but several variables, including cell type, cellular microenvironment, and genetic background, could affect the outcome [38, 39]. CDKN2A (p16) is generally understood to be an apoptosis regulatory gene, which may be involved in the pathogenesis and development of endometriosis [40]. In women with endometriosis, the altered p16 expressions has been evidenced in eutopic endometrium [41]. Stromal p16 level is a representative discovery in endometrial polyps [42]. In benign lesions, overexpression of p16 suppresses cell proliferation, keeping cells from malignant transformation [43]. We found that hucMSC-Ex downregulated the increased CDKN2A induced by hypoxia in EECs. CDKN2A expression could be negatively modulated by miR-663a. Moreover, overexpression of miR-663a in hypoxia-induced EECs increased antiapoptotic protein Bcl-2, as well as increased epithelial marker E-cadherin. Therefore, hucMSC-Ex exerted a protective function in hypoxia-induced EECs injury, which may be related to the regulation of the miR-663a/CDKN2A axis.

Studies have observed that exosomes can carry functional RNAs, miRNAs, and proteins among cells [44, 45]. Exosomes derived from MSCs inhibit apoptosis through miRNA regulating signaling pathway in ESCs, which could effectively improve endometrial repair [11]. Although we found that hucMCS-Ex could improve hypoxia-induced cell viability and inhibit apoptosis in EECs, it may play a role in regulating the miR-663a/CDKN2A axis. But whether miR-663a also acts on EECs cells through hucMCS-Ex as a vector requires further experimental investigation. In addition, more experiments are needed to further explore the role and mechanism of miR-663a and CDKN2A in hypoxia-induced proliferation, migration, and apoptosis of EECs.

## 5. Conclusion

In conclusion, hucMSC-Ex treatment upregulated the expression of miR-663 in EECs that were downregulated by hypoxia, and miR-663 targeted and regulated the expression of CDKN2A. These results indicate that the protective function of hucMSC-Ex in hypoxia-induced EECs injury may be related to regulation of the miR-663a/CDKN2A axis. This research may provide new insights into thin endometrium treatment.

## Figures and Tables

**Figure 1:** Characterization of hucMSCs. (a)–(f) The surface antigens (CD73, CD90, CD105, CD14, CD34, and CD45) of hucMSCs were detected by flow cytometry.

**Figure 2:** Characterization of hucMSC-Ex. (a) CD63 and TSG101 protein expression in hucMSC-Ex were measured with western blot. (b) Exosomes from the culture medium of hucMSCs were observed by transmission electron microscopic (TEM). The scale bar represents 100 nm. (c) Nanoparticle tracking analysis (NTA) data exhibited the average diameter and particle number of hucMSC-Ex.

**Figure 3:** HucMSC-Ex promoted EECs survival under hypoxic condition. (a–d) The protein expression of epithelial marker E-cadherin, as well as hypoxia-related proteins (VEGF and av*β*3), was monitored by western blot. EECs were cultured for the indicated times (1, 4, 8, 16, and 24 h) under hypoxic condition. (e) EECs were maintained under normoxic (normal group), hypoxic (hypoxia group), or hypoxic condition for 4 h followed by cocultured with PKH67-labeled hucMSC-Ex for 24 h (hypoxia+hucMSC-Ex). PKH67-labeled hucMSC-Ex within EECs were analyzed, and the scale bar represents 200 *μ*m. (f) Cell viability of EECs was detected by Cell Counting Kit-8 (CCK-8), ^∗∗∗∗^*P* < 0.0001 and ^∗∗^*P* < 0.01 versus normal group, ^#^*P* < 0.05 and ^##^*P* < 0.01 versus hypoxia group.

**Figure 4:** HucMSC-Ex inhibited hypoxia induced apoptosis, migration, and EMT of EECs. (a,b) Cell apoptosis of EECs was analyzed by flow cytometry. (c,d) Cell migration of EECs was assessed by wound healing assay. (e–j) Apoptosis-related proteins (Bax, cleaved-caspase3, P53, and Bcl-2), and EMT-related proteins (N-cadherin and E-cadherin) were analyzed with western blot. ^∗^*P* < 0.05, ^∗∗^*P* < 0.01, ^∗∗∗^*P* < 0.001, ^∗∗∗∗^*P* < 0.0001. Data are expressed as mean ± SD. *n* = 3.

**Figure 5:** HucMSC-Ex increased miR-663a in hypoxia-treated EECs, and miR-663a negatively regulated CDKN2A expression. (a) DEmiRNA in the hypoxia, normal, and hypoxia+hucMSC-Ex groups was visualized by Volcano plot. Red and blue dots showed expressions increased and decreased miRNAs, respectively. (b) Profiling of miRNAs in the normal, hypoxia, and hypoxia+hucMSC-Ex groups was displayed by heat map. Blue color indicated relative low level and red color indicated relative high level in comparison with the normal group (left panel). (c) The miR-663a level in EECs was detected by qRT-PCR. (d) The target sequence of miR-663a and CDKN2A was predicted by online website TargentScanHuman (https://www.targetscan.org/vert_80/). (e) qRT-PCR was carried out for detecting the mRNA levels of CDKN2A in EECs. (f) The miR-663a level in hypoxia-induced EECs transfected by miR-663a mimics was detected by qRT-PCR. (g–l) The protein expression of CDKN2A (p16INK4a), E-cadherin, N-cadherin, Bax, and Bcl-2 in hypoxia-induced EECs transfected with miR-663a mimics or NC was detected using western blot. ^∗∗∗^*P* < 0.001, ^∗∗∗∗^*P* < 0.0001. Data are expressed as mean ± SD. *n* = 3.

**Table 1:** List of primer sequences for qRT-PCR.

Gene name	Primer sequence (5′ to 3′)
Hsa-miR-663a	F: CTCAACTGGTGTCGTGGA
Hsa-miR-663a	R: GCCGAGAGGCGGGGCGCCGCGG
Hsa-U6	F: GCTTCGGCAGCACATATACT
Hsa-U6	R: ACGCTTCACGAATTTGCGTG
CDKN2A	F: CCACGGCGCGGAGCCCAA
CDKN2A	R: GCAGCACCACCAGCGTGTCCA
GAPDH	F: TCAAGATCATCAGCAATGCC
GAPDH	R: CGATACCAAAGTTGTCATGGA

## Data Availability

The data used to support the findings of this study are available from the corresponding author upon request.

## Abbreviations

hucMSCs: Human umbilical cord mesenchymal stem cells
BMSCs: Bone marrow mesenchymal stem cells
hucMSC-Ex: Human umbilical cord mesenchymal stem cell-derived exosome
EECs: Endometrial epithelial cells
OGD/R: Oxygen and glucose deprivation/reoxygenation
TEM: Transmission electron microscopy
NTA: Nanoparticle tracking analysis
CCK-8: Cell counting kit-8
RT-qPCR: Real time-quantitative polymerase chain reaction
ESCs: Endometrial stromal cells
EMT: Epithelial-mesenchymal transition
miRNAs: MicroRNAs
DAPI: 4′, 6-diamidino-2-phenylindole
WB: Western blot
IF: Immunofluorescent
SD: Standard deviation.
